The article "Chondroprotective Effects of Gubitong Recipe via Inhibiting Excessive Mitophagy of Chondrocytes" was published in 2022. Journal: Evid Based Complement Alternat Med.

# Chondroprotective Effects of Gubitong Recipe via Inhibiting Excessive Mitophagy of Chondrocytes

**DOI:** 10.1155/2022/8922021

**Published:** 2022-08-01

**Authors:** Xin-bo Yu, Guang-yao Chen, Li Zhou, Li-li Deng, Wei-jiang Song, Jia-qi Chen, Qian He, Cai-qin Xu, Jing Luo, Qing-wen Tao

**Affiliations:** ^1^Graduate School, Beijing University of Chinese Medicine, Beijing 100029, China; ^2^Traditional Chinese Medicine Department of Rheumatology, China-Japan Friendship Hospital, Beijing 100029, China; ^3^Rehabilitation Department, Qingdao Huangdao District No. 2 Chinese Medicine Hospital, Qingdao 266400, China; ^4^Traditional Chinese Medicine Department, Peking University Third Hospital, Beijing, China; ^5^Beijing Key Laboratory of Immune Inflammatory Disease, China-Japan Friendship Hospital, Beijing 100029, China

## Abstract

**Objective:**

Osteoarthritis (OA) is the most common degenerative joint disorder and a leading cause of disability. A previous randomized controlled trial has shown that Gubitong (GBT) recipe can improve OA-related symptoms and articular function without noticeable side effects. However, the underlying mechanisms remain unclear. This study aims to explore the therapeutic mechanisms of the GBT recipe for OA through in vivo and in vitro experiments.

**Methods:**

Rats of the OA model were established by Hulth surgery and intervened with the GBT recipe and then were subjected to pathological assessment of the cartilage. Matrix metalloproteinase 13 (MMP-13) expression in cartilage tissues was assessed by immunohistochemical staining. Chondrocytes were isolated from sucking rats and stimulated with LPS to establish an in vitro model. After intervened by water extraction of the GBT recipe, the fluorescent signal of Mtphagy Dye and mitochondrial membrane potential (Δ*ψ*m) were detected to determine the states of mitophagy and mitochondrial dynamics of chondrocytes in vitro, respectively. Western blot test was used to detect levels of proteins related to catabolism of the cartilage matrix, mitophagy, and PI3K/AKT pathway.

**Results:**

In in vivo experiments, the GBT recipe can effectively inhibit the cartilage degeneration of chondrocytes in OA rats, as well as markedly suppress the expression of MMP-13. In vitro experiments on LPS-induced chondrocytes exhibited increase in mitochondrial depolarization and excessive mitophagy, and the GBT recipe can alleviate these changes. LPS-stimulated chondrocytes showed increases in MMP-13, PINK1, and Parkin in cell lysates and LC3II/LC3I ratio in the mitochondrial fraction, and the GBT recipe can inhibit these increases in a dose-dependent manner. Moreover, the GBT recipe can attenuate the abnormal activation of PI3K/AKT pathway induced by LPS.

The article "Chondroprotective Effects of Gubitong Recipe via Inhibiting Excessive Mitophagy of Chondrocytes" was published in 2022. Journal: Evid Based Complement Alternat Med.

**Conclusion:**

The GBT recipe exhibits chondroprotective effects through inhibiting excessive mitophagy of chondrocytes, which may be associated with its inhibitory effect on the abnormal activation of PI3K/AKT pathway.

## 1. Introduction

Osteoarthritis (OA) is a common and disabling condition characterized by degeneration of articular cartilage [1]. With an aging population and increasing rates of obesity, OA is becoming more prevalent than in previous decades [2]. A study based on the National Health Interview Survey (NHIS) of the United States showed that 22.7% of the adult population had at least one joint affected by OA and the incidence increased to 49.6% for those beyond the age of 65 [3]. Patients with OA often have pain, morning stiffness, crepitus on joint motion, and even instability or physical disability of joint, which impair quality of life and lead to a considerable socioeconomic burden [4].

Articular cartilage consists of a rich extracellular matrix (ECM) with a sparse dispersion of chondrocytes [5]. Adult articular cartilage is devoid of both innervation and vascularization, and chondrocytes are responsible for the anabolism and catabolism balance of ECM. Injured chondrocytes in osteoarthritic cartilage manufacture less ECM than usual, contributing to the irreversible degenerative process of OA [6, 7]. The anabolic and catabolic processes of chondrocytes are intimately linked to mitochondrial functions [8]. Mitophagy, a selective form of autophagy that removes damaged or excessive mitochondria, is essential in maintaining cellular energy homeostasis and function [9]. However, excessive mitophagy can result in excessive mitochondrial oxidative stress and mitochondrial functions decline, leading to chondrocytes degeneration and cartilage destruction, and finally to OA [10, 11].

Current management for OA focuses on relieving pain and inflammation, alleviating cartilage degeneration, and improving articular function [12]. Commonly, the treatment of OA includes pharmacological therapies, nonpharmacological therapies, and joint replacement surgery [13–15]. Nonsteroidal anti-inflammatory drugs (NSAIDs) are the most commonly recommended drugs for OA [15]. However, long-term applications of NSAIDs in patients with OA are controversial due to the gastrointestinal and cardiovascular side effects [16,17]. There are no specific and efficacious disease-modifying drugs for OA yet [14]. Thus, it is desirable to develop a more effective and safer drug.

Traditional Chinese medicine (TCM) has been used to treat a variety of medical conditions including OA in China for thousands of years. Recently, some randomized controlled trials (RCTs) have demonstrated the therapeutic effect and safety of herbal medicine in treating OA [16–19]. Gubitong (GBT) recipe, a TCM prescription consisting of eight herbs, has also shown its therapeutic potential for patients with OA in a previous RCT [19]. However, the underlying mechanisms remain unclear. This study aims to explore the therapeutic mechanisms of the GBT recipe for OA through in vivo and in vitro experiments.

The article "Chondroprotective Effects of Gubitong Recipe via Inhibiting Excessive Mitophagy of Chondrocytes" was published in 2022. Journal: Evid Based Complement Alternat Med.

## 2. Materials and Methods

### 2.1. Reagents and Antibodies

0.25% Trypsin-EDTA, DMEM medium, phosphate-buffered saline (PBS), fetal bovine serum (FBS), and collagenase II were purchased from Gibco. Lipopolysaccharides (LPS), penicillin-streptomycin and poly-L-lysine, and Triton X-100 were purchased from Sigma. Electrochemiluminescence (ECL) luminous fluid and polyvinylidene difluoride (PVDF) membranes were purchased from Millipore. Animal-free blocking solution was purchased from Cell Signaling. Mitochondrial extraction kit, RIPA lysis buffer, phenylmethanesulfonyl fluoride (PMSF), protein phosphatase inhibitor, Tween-20, and EDTA-Na_2_ were purchased from Solarbio Life Sciences. SDS-PAGE running buffer powder, Tris-buffered saline (TBS) powder, and SDS-PAGE transfer buffer powder were purchased from Servicebio. A fluorescent mounting medium with DAPI (4,6-diamidino-2-phenylindole) was purchased from Zhongshan Jingqiao Biotechnology. Mtphagy Dye was purchased from Dojindo Laboratories.

Anticollagen II antibody (ab34712) and anti-MMP-13 antibody (ab39012) were purchased from Abcam. Anti-AKT antibody (4691S) and anti-phospho-AKT (Ser473) antibody (4060S) were purchased from Cell Signaling Technology. Anti-Parkin antibody (sc-32282) was purchased from Santa Cruz. Anti-PINK1 antibody (A11435), anti-LC3B antibody (A19665), anti-COX IV antibody (A6564), and anti-PI3K p85 antibody (A4992) were purchased from ABclonal. Anti-phospho-PI3K antibody (YP0224) was purchased from Immunoway. *β*-Actin antibody (TA-09), horseradish peroxidase (HRP)-conjugated goat anti-mouse IgG (ZB-5305), HRP-conjugated goat anti-rabbit IgG (ZB-2301), and Alexa Fluor 488-conjugated goat anti-rabbit IgG (H + L) (ZF-0511) were purchased from Zhongshan Jingqiao Biotechnology.

### 2.2. Preparation of GBT Recipe

GBT recipe, which consists of Rhizoma Drynariae 20 g, Epimedii Folium 15 g, Fructus Psoraleae 15 g, Cortex Eucommiae 30 g, Rhizoma Cibotii 30 g, Rhizoma Bolbostemmae 20 g, Caulis Sinomenii 30 g, and Caulis Spatholobi 30 g, was purchased from TCM Pharmacy of China-Japan Friendship Hospital. Each drug of the GBT recipe was validated by an herbal medicinal botanist from the Beijing University of Chinese Medicine. Drugs were soaked in a 10-fold volume of distilled water for 4 hours. After 1 hour of decoction, the suspension of the GBT recipe was filtered three times. The filtered decoction was concentrated under reduced pressure on a rotary evaporator. The concentrated solution was refrigerated for 12 hours at 4°C and then centrifuged to obtain a suspension. After boiling the final supernatant, dehydrated alcohol was gently added with quick agitation until the concentration reached 75% alcohol (v/v). The filtrate was then centrifuged after cooling and decompressed into a paste having a relative density of 1.25 g/ml (w/v). The paste was then lyophilized under vacuum.

The article "Chondroprotective Effects of Gubitong Recipe via Inhibiting Excessive Mitophagy of Chondrocytes" was published in 2022. Journal: Evid Based Complement Alternat Med.

### 2.3. Liquid Chromatography-Mass Spectrometry Analysis

Reversed-phase chromatography was performed using a Nexera High-Performance Liquid Chromatograph (Japan Shimadzu Co., Ltd) coupled to the SCIEX 5600 Triple-TOF Mass Spectrometer (Sciex, Toronto, Canada). The samples were eluted on HSS T3 C18 analytical column (2.1 × 100 mm, 1.8 *μ*m) with a 30 min gradient at a flow rate of 0.3 mL/min. The two mobile phases consisted of buffer A (0.1% formic acid/99.9% H_2_O) and buffer B (99.9% acetonitrile/0.1% formic acid) and operated under the following program: 0–5 min, 15%–15% B; 5–13 min, 15%-16% B; 13–17 min, 16%–16% B; 17–20 min, 16%-17% B; 20–26 min, 11%–95% B; 26-27 min, 95%–15% B; and 27–30 min, 15%-15% B. The scan mode for high-resolution mass spectrometry acquisition was full-scan/dd-MS2 mode, and data were acquired in the m/z range 100–1,500.

### 2.4. Animals Feeding

Seven-week-old male Sprague–Dawley (SD) rats were purchased from SPF (Beijing) Biotechnology Co., Ltd. The rats were raised in a clean-grade animal room with a temperature of 23 ± 2°C and a humidity of 50 ± 10% in the Experimental Animal Center of China-Japan Friendship Hospital. All animal experiment procedures were approved by the Animal Care and Welfare Committee of China-Japan Friendship Hospital (No. zryhyy21-21-05-09). After 7 days of adaptive feeding, the rats were randomly divided into four groups, including blank control group, model group, GBT recipe group, and glucosamine sulfate group, according to the random digital table method.

### 2.5. OA Model Preparation and Intervention

The rats were anesthetized by isoflurane inhalation. After fur was shaven off, the skins of the left keen joint were sterilized with iodophor. A surgical knife was used to transversely incise the skin of the left keen joint and patellar ligament. After the medial collateral ligament was severed and meniscus was drawn, anterior and posterior cruciate ligaments were severed. The incision was sutured layer by layer after a drawer test was positive. Penicillin (200,000 units) was injected into each rat that underwent surgery for successive three days to avoid infection. A typical daily dose of GBT recipe and glucosamine sulfate in the treatment of OA was 190 g and 1440 mg, and a human reference weight of an adult is 60 kg. Thus, the dose of GBT recipe and glucosamine to be administered is 3.2 g/kg and 1.7 mg/kg for an adult. According to the guide for dose conversion between animals and humans, the dose for rats is 6.3 times that of humans [20]. Based on this, the dose of GBT recipe in rats should roughly be 20.2 g/kg/day, and the dose of glucosamine sulfate should roughly be 150 mg/kg/d. Beginning on the 4th day following surgery, glucosamine sulfate and GBT recipe were given to rats once a day. Rats were sacrificed by inhalation of CO_2_ (compressed CO_2_ gas cylinder) at 4 weeks after administration. The left knee joint was separated for pathological assessment.

The article "Chondroprotective Effects of Gubitong Recipe via Inhibiting Excessive Mitophagy of Chondrocytes" was published in 2022. Journal: Evid Based Complement Alternat Med.

### 2.6. Pathological Assessment

The knee joints of rats were fixed with 4% paraformaldehyde for 72 hours and decalcified in 10% ethylenediaminetetraacetic acid-Na_2_ (EDTA-Na_2_) for 6 weeks. The tissues were dehydrated, embedded, and sliced into 4 *μ*m sections. The sections were then stained with hematoxylin and eosin (HE) and safranin O-fast green (SCO) staining for histological examination. Mankin's scoring method was used to evaluate the articular cartilage degeneration [21]. Each section was assessed by a well-trained researcher without being informed of the grouping.

### 2.7. Immunohistochemistry

The paraffin-embedded tissues were used for the immunohistochemical analysis of MMP-13 expression in the articular cartilage of rats. In brief, after the slides were incubated with a blocking serum for 30 min, they were blotted and then overlaid with the primary antibody against MMP-13 for 2 h at room temperature. Subsequently, biotinylated secondary antibodies were added into the sections, followed by a peroxidase-labeled streptavidin-biotin staining technique. Finally, the samples were observed under a light microscope. The images from the immunohistochemistry samples were quantified using Image-Pro Plus software.

### 2.8. Isolation and Culture of Chondrocytes

Five-day sucking rats were sacrificed by inhalation of CO_2_ (compressed CO_2_ gas cylinder). The knee joint cartilage was isolated in a sterile environment and digested using 0.25% trypsin for 1 hour. The cartilage was neutralized with DMEM containing 10% FBS and washed three times with PBS. After digested with 2 mg/ml type II collagenase for 6 hours, the joint cartilage was filtered with a 100-mesh stainless steel screen to prepare for chondrocytes suspensions. The suspensions were centrifuged to collect chondrocytes. Chondrocytes were seeded in a DMEM medium with 10% FBS, 50 U/ml penicillin, and 50 *μ*g/ml streptomycin and cultured on polylysine-coated dishes. A second or third generation of chondrocytes was used for cell experiments.

The article "Chondroprotective Effects of Gubitong Recipe via Inhibiting Excessive Mitophagy of Chondrocytes" was published in 2022. Journal: Evid Based Complement Alternat Med.

### 2.9. MTS Assay

MTS assay was used to evaluate the effect of the GBT recipe on the vitality of chondrocytes. 1 × 10^4^ chondrocytes were seeded into 96-well culture plates. After cells were completely adherent, the culture medium was discarded and the cells were treated with different concentrations of the GBT recipe for 12 hours. Then, the cells were incubated for 4 hours in a DMEM medium. Subsequently, 20 *μ*L MTS reagent was added to the cells, followed by another 20 min of incubation. A microplate reader was used to detect absorbance at a wavelength of 490 nm.

### 2.10. Cell Culture and Treatment

Chondrocytes were cultured in a DMEM medium containing 10% FBS, 50 U/ml penicillin, and 50 *μ*g/ml streptomycin. Cells were subcultured every 2–3 days at 37°C in a humidified 5% CO_2_ environment. Chondrocytes were pretreated with DEX (100 nmol/ml) or different GBT recipe concentrations (50, 100, and 200 ug/ml) for 1 hour, and then, LPS (100 ng/ml) was added for 12 hours.

### 2.11. Mitochondrial Isolation

Chondrocyte mitochondria were isolated using a mitochondrial extraction kit. Chondrocytes were homogenized using a Dounce-type glass homogenizer in precold lysis buffer and centrifuged at 1000 g for 10 minutes. The mitochondria were then pelleted by centrifuging the crude supernatant for 10 minutes at 12,000 g. Precipitates were resuspended in 0.5 mL wash buffer and centrifuged at 1000 g for 5 min. Mitochondria were ultimately separated from the supernatant by centrifugation at 12,000 g for 10 minutes at 4°C.

### 2.12. Reverse Transcription and Quantitative Real-Time PCR

RNA was extracted from chondrocytes and SW1353 cells using the column-based HiPure Total RNA Mini Kit. Then, RNA concentration and purity were measured. 1 ug RNA was reverse transcribed into cDNA using a reverse transcription system. The qRT-PCR was performed in a total volume of 20 *μ*l, with 2 *μ*l of cDNA, 10 *μ*l of SYBR Green qPCR Mix, and 2 *μ*M of the forward and reverse primers in each tube. The CT values of each sample were acquired after the end of the reaction.

### 2.13. Western Blot Analysis

The samples were lysed by RIPA buffer with 1% PMSF and 1% phosphatase inhibitors on ice for 30 min. After centrifugation at 10,000 g for 10 minutes at 4°C, the supernatant was collected. The bicinchoninic acid (BCA) method was used to quantify the protein content. Protein samples were boiled after the addition of loading buffer, and 40 *μ*g of each protein sample was loaded onto the SDS-PAGE gels. The protein was separated by SDS-PAG electrophoresis (SDS-PAGE) and transferred to PVDF membrane (70 v, 55 min). PVDF membrane was then blocked with 5% nonfat milk powder for 1 hour at room temperature. The membranes were then incubated with primary antibodies overnight at 4°C. After washing with TBS containing 0.05% Tween-20 (TBST), membranes were incubated with secondary antibodies for 2 hours at room temperature. The protein samples were visualized using a chemiluminescence machine (Bio-Rad, USA). The primary antibodies associated parameters are listed in Table 1.

The article "Chondroprotective Effects of Gubitong Recipe via Inhibiting Excessive Mitophagy of Chondrocytes" was published in 2022. Journal: Evid Based Complement Alternat Med.

### 2.14. Immunofluorescence Staining

Chondrocytes were inoculated on a 48-well plate and cultured for 24 hours. The culture medium was discarded after completion and the plate was washed with PBS at 37°C. The cells were fixed for 15 minutes at room temperature with 4% paraformaldehyde and then permeabilized for 5 minutes with 0.1% Triton X-100/PBS. After washing three times with PBS, cells were blocked for 1 hour with an animal-free blocking solution. Then, cells were incubated with antibodies against type II collagen (1 : 100 dilution) overnight at 4°C. Cells were washed three times with PBS and incubated with fluorescein (FITC)-conjugated goat anti-rabbit IgG (1 : 50 dilution) at room temperature for 1 hour. After the cells were washed three times with PBS, the nuclei were stained with DAPI and observed under an inverted fluorescence microscope.

### 2.15. Mitophagy Assay

A Mitophagy Detection Kit (Dojindo Molecular Technologies) was used to detect mitophagy [22]. The chondrocytes were washed twice with DMEM and incubated with 100 nM Mtphagy Dye diluted in DMEM for 30 min at 37 °C. After incubation, cells were washed twice with DMEM and continued to be incubated for another 1 h in the previous culture conditions. After mitochondrial staining, the dye was immobilized and fluorescence intensity varied according to pH value. In mitochondrial-lysosome fusion, Mtphagy Dye displayed higher fluorescence intensity, indicating mitophagy. The level of mitophagy was defined by the area of Mtphagy Dye per cell.

### 2.16. Flow Cytometry

In the measurement of type II collagen, chondrocytes were fixed and incubated with type II collagen primary antibody (1 : 50 dilution) for 1 hour after discarding the culture supernatant. Subsequently, the cells were incubated with fluorescein isothiocyanate (FITC)-conjugated anti-rabbit antibody for 30 minutes and then detected by flow cytometry. Mitochondrial membrane potential was measured using a mitochondrial membrane potential assay kit with JC-1 according to the manufacturer's protocol.

The article "Chondroprotective Effects of Gubitong Recipe via Inhibiting Excessive Mitophagy of Chondrocytes" was published in 2022. Journal: Evid Based Complement Alternat Med.

### 2.17. Statistical Analysis

Statistical analysis was performed using SPSS 19 statistical package. Student's *t*-test was used to detect the statistically significant differences between experimental groups. Data were presented as mean ± standard deviation; a two-sided *p* < 0.05 was considered statistically significant.

## 3. Results

### 3.1. Quality Control of GBT Recipe Extraction

Representative components of each herb in the GBT recipe were selected according to the Chinese Pharmacopoeia (2020 edition) and relevant literature [23]. There were nine representative components in GBT recipe including naringin (from Rhizoma Drynariae), icariin (from Epimedii Folium), psoralen (from Fructus Psoraleae), pinoresinol diglucoside (from Cortex Eucommiae), protocatechuic acid (from Rhizoma Cibotii), tubeimoside I (from Rhizoma Bolbostemmae), sinomenine (from Caulis Sinomenii), and catechin and epicatechin (from Caulis Spatholobi). Liquid chromatography coupled with mass spectrometry (LC-MS) results showed that all the nine components were present in GBT recipe extraction (Figure 1), and the detailed information is shown in Table 2.

### 3.2. Protective Effects of GBT Recipe on Joints Cartilage of OA Rats

Pathological changes in knee joint cartilage in each group are shown in Figure 2. Compared with the blank control group, the cartilage in the model group exhibited a successful establishment of the OA model and a significantly higher Mankin's score: the articular cartilage surface layer was fiberized, chondrocytes were severely proliferated and hypertrophied, cell lamination was completely disordered, and cytoplasmic vacuolization resulting from apoptotic cells was increased (Figures 2(a), 2(b), 2(e), and 2(f)). After GBT recipe treatment, cartilage lesion and matrix degradation were well ameliorated (Figures 2(c) and 2(g)). Meanwhile, the improvement of cartilage degeneration in the glucosamine sulfate group was inferior to that in the GBT recipe group (Figures 2(d) and 2(h)).

### 3.3. Effect of GBT Recipe on MMP-13 in the Articular Cartilage

The results of immunohistochemistry showed that MMP-13 increased in cartilage of the OA model group (Figures 3(a) and 3(b)). The GBT recipe and glucosamine sulfate could reduce the abnormal increase caused by OA, and the GBT recipe was more effective than glucosamine sulfate (*p* < 0.05) (Figures 3(c) and 3(d)).

### 3.4. Identification of Chondrocytes

The identification of chondrocytes by type II collagen expression is shown in Figure 4. The immunofluorescence analysis showed that nearly all chondrocytes were positive for type II collagen (Figures 4(a), 4(b), and 4(c)). The proportion of type II collagen-positive chondrocytes was further assessed by flow cytometry. The results indicated that the proportion of chondrocytes expressing type II collagen was 98 ± 1.1% (*n* = 3), and none for SW1353 cell-expressed type II collagen (Figures 4(d) and 4(e)). The qRT-PCR results demonstrated that chondrocytes expressed large amounts of type II collagen mRNA but the mRNA expression of type II collagen was not detectable in SW1353 cells (Figure 4(f)).

The article "Chondroprotective Effects of Gubitong Recipe via Inhibiting Excessive Mitophagy of Chondrocytes" was published in 2022. Journal: Evid Based Complement Alternat Med.

### 3.5. Effects of GBT Recipe on Chondrocytes Viability

To evaluate the effects of the GBT recipe on chondrocytes, the chondrocytes were incubated in a medium containing various concentrations of the GBT recipe (0, 50, 100, 150, 200, and 250 *μ*g/ml) for 12 hours. MTS assay was performed to evaluate the viability of chondrocytes after treating with the GBT recipe. There was no significant effect on chondrocytes viability among concentrations of 0, 50, 100, 150, and 200 *μ*g/ml. The chondrocytes viability was significantly decreased at the concentration of 250 *μ*g/ml (Figure 5). These results demonstrated that 200 ug/ml was the maximum intervention concentration of the GBT recipe for chondrocytes. Therefore, 50 *μ*g/ml, 100 *μ*g/ml, and 200 *μ*g/ml were chosen as low, intermediate, and high concentrations of the GBT recipe, respectively.

### 3.6. Effects of GBT Recipe on LPS-Induced MMP-13 Expression in Chondrocytes

Western blot and RT-PCR analyses showed that compared with LPS-free chondrocytes, LPS-induced chondrocytes had an increased expression of MMP-13 at the gene and protein levels. However, these changes in LPS-induced chondrocytes were reversed by the GBT recipe and DEX, and the GBT recipe showed a dose-dependent effect (Figure 6).

### 3.7. Effects of GBT Recipe on LPS-Induced Mitophagy in Chondrocytes

Mitophagy was detected using Mtphagy Dye. Compared with unstimulated chondrocytes, a significant increase in the fluorescent signal of Mtphagy Dye was detected in LPS-stimulated chondrocytes (Figures 7(a) and 7(b)). These changes could be suppressed by 200 *μ*g/ml GBT recipe and 100 nmol/ml DEX (Figures 7(c) and 7(d)).

### 3.8. Effects of GBT Recipe on LPS-Induced Mitochondrial Dynamics in Chondrocytes

We used the JC-1 assay to measure mitochondrial membrane potential (Δ*ψ*m) changes to see if LPS-induced mitophagy affects mitochondrial dynamics. LPS treatment significantly increased mitochondrial depolarization, as evidenced by a decrease in the red/green fluorescence intensity ratio (Figures 8(a) and 8(b)). 200 *μ*g/ml GBT recipe and 100 nmol/ml DEX stabilize the mitochondrial membrane potential (Δ*ψ*m) significantly (Figures 8(c) and 8(d)).

### 3.9. Effects of GBT Recipe on Protein Expression Associated with Chondrocyte Mitophagy in Chondrocytes

Western blot analysis showed that LPS elevated the ratio of LC3II and LC3I (LC3II/LC3I) in mitochondria of chondrocytes. Meanwhile, compared with LPS-free chondrocytes, LPS-induced chondrocytes had an increased expression of PINK1 and Parkin. However, these changes in LPS-induced chondrocytes were reversed by the GBT recipe and DEX, and the GBT recipe showed a dose-dependent effect (Figure 9).

The article "Chondroprotective Effects of Gubitong Recipe via Inhibiting Excessive Mitophagy of Chondrocytes" was published in 2022. Journal: Evid Based Complement Alternat Med.

### 3.10. Effects of GBT Recipe on PI3K/AKT Signaling Pathway in Chondrocytes

Western blot revealed that the levels of PI3K and AKT proteins in LPS-induced chondrocytes were not changed compared with LPS-free chondrocytes, but the expression of p-PI3K and p-AKT was increased, suggesting that LPS abnormally activated the PI3K/AKT signaling pathway in chondrocyte (Figure 10). In addition, the phosphorylation levels of PI3K and AKT were reversed by the GBT recipe in a dose-dependent manner.

## 4. Discussion

Chondrocytes are the only cell type in cartilage and numerous studies have shown that OA often occurs with chondrocyte senescence and apoptosis [6, 24, 25]. During the pathologic process of OA, the capacity of chondrocytes to synthesize cartilage matrix was greatly reduced and large amounts of proteolytic enzymes were released, such as MMP-13, causing damage to the cartilage matrix [26]. Thus, improving the function of OA chondrocytes may be a target in treating OA [27].

Our study showed that the GBT recipe can effectively suppress the cartilage degeneration and apoptosis of the chondrocytes in the OA rat model. This was consistent with a previous study [28]. We found an increased expression of MMP-13 in the OA rat model by immunohistochemistry. MMP-13 was a hallmark of chondrocyte senescence and apoptosis and thus considered an important cause of the cartilage degeneration [29–31]. The intragastric administration of the GBT recipe can effectively reverse the high expression of MMP-13 in cartilage tissue of the OA rat model, which may indicate the therapeutic potential and mechanism of the GBT recipe for OA.

To further explore the therapeutic mechanisms of the GBT recipe for OA, we established an OA cell model by LPS-induced chondrocytes in vitro. The results showed that the mRNA and protein expressions of MMP-13 were significantly increased in LPS-induced chondrocytes and the GBT recipe can reverse this phenomenon in a dose-dependent manner. This suggests that the GBT recipe can promote chondroprotection by inhibiting the expression of MMP-13 in inflammatory chondrocytes.

JC-1 has been widely used to detect mitochondrial membrane potential as a fluorescent probe [32, 33]. The JC-1 dye accumulates in mitochondria in a potential-dependent manner, which is usually indicated by a shift in fluorescence emission from green (535 nm) to red (595 nm). JC-1 forms aggregates with intense red fluorescence in healthy mitochondria with high ΔΨm, and monomers with green fluorescence when ΔΨm diminishes (depolarization) [34]. When the mitochondria are damaged, the mitochondrial membrane potential decrease in cells, the J-aggregate (red fluorescence) declines and the JC-1 monomer (green fluorescence) increases. The mitophagy detection kit is a common detection method for mitophagy after mitochondrial staining; the dye is immobilized and fluorescence intensity varies according to pH value [35, 36]. In mitochondrial-lysosome fusion, Mtphagy Dye displays higher fluorescence intensity, indicating mitophagy.

The article "Chondroprotective Effects of Gubitong Recipe via Inhibiting Excessive Mitophagy of Chondrocytes" was published in 2022. Journal: Evid Based Complement Alternat Med.

Our study showed that there was a decrease in the red/green fluorescence intensity ratio in LPS-induced chondrocytes, which indicated that the mitochondria membrane potential was depolarized and the mitochondrial function was impaired. Concurrently, the level of mitophagy in inflammatory chondrocytes was significantly elevated by analyzing the fluorescence intensity of Mtphagy Dye. These results revealed that excessive mitophagy was induced by LPS stimulation causing mitochondrial dysfunction. In further chondrocyte experiments, we found that the expression of the following two key molecules in mitophagy regulation was much higher in the LPS group than in the control group: Parkin and PINK1, and the LC3II/LC3I ratio. These results corroborate the excessive mitophagy in LPS-induced chondrocytes.

ROS are primarily generated in mitochondria, and mitochondrial abnormalities can induce ROS overproduction, leading to abnormal activation of the NF*κ*B signaling pathway, eventually promoting MMPs expression [37–40]. The GBT recipe and the positive control drug (Dex) can inhibit the mitochondrial depolarization and the expression of mitophagy-related proteins and thus alleviate excessive mitophagy. Overall, inhibiting the excessive mitophagy of inflammatory chondrocytes may be the key mechanism by which the GBT recipe protects chondrocytes.

Previous studies have demonstrated that the PI3K/AKT pathway is associated with the inflammatory response, apoptosis, and autophagy of chondrocytes and thus is closely related to the development of OA [41–43]. The inhibition of the PI3K/AKT pathway can reduce cartilage degeneration by regulating the expression of multiple downstream targets. Hence, the PI3K/AKT pathway is considered a potential therapeutic target in treating OA [44]. In our in vitro experiments, chondrocytes showed elevated levels of phosphorylated PI3K and phosphorylated AKT after LPS stimulation. Meanwhile, the GBT recipe reduced these changes in LPS-induced chondrocytes, suggesting that the GBT recipe can inhibit the abnormal activation of the PI3K/AKT pathway, which may be associated with its chondroprotective effects and need further research in the future.

The article "Chondroprotective Effects of Gubitong Recipe via Inhibiting Excessive Mitophagy of Chondrocytes" was published in 2022. Journal: Evid Based Complement Alternat Med.

In conclusion, the GBT recipe showed chondroprotective effects on OA rats and rat chondrocytes stimulated by LPS. The chondroprotective effects may be associated with the inhibition of excessive mitophagy and abnormal activation of the PI3K/AKT pathway. Taken together, we suggest that the GBT recipe can be an effective alternative therapy in preventing and treating OA. However, we did not explore the effect of the GBT recipe in synovitis and human OA chondrocytes in this experiment. More studies are still needed to further investigate and validate the protective effects of the GBT recipe for OA.

## Figures and Tables

**Figure 1:** Total ion chromatography (TIC) on positive and negative and extraction ion chromatography of GBT recipe.

**Figure 2:** Pathological changes of cartilage. (a, e) Blank control group of hematoxylin-eosin (HE) staining and safranin O/fast green (S-O) staining. (b, f) Model group of HE and S-O staining. (c, g) GBT recipe group of HE and SCO staining. (d, h) Glucosamine sulfate group of HE and S-O staining. (I) Mankin's score of each group. Data were presented as mean ± standard deviation (^*∗*^*p* < 0.05 compared with the blank control group; ^#^*p* < 0.05 compared with the OA model group). (a) Blank control group; (b) model group; (c) GBT recipe group; (d) glucosamine sulfate group.

**Figure 3:** (a) Immunohistochemistry (IHC) for MMP-13 in cartilage from blank control group rat knee joints. (b) IHC for MMP-13 in the cartilage from the OA model group rat knee joints. (c) IHC for MMP-13 in the cartilage from the GBT recipe group rat knee joints. (d) IHC for MMP-13 in the cartilage from the glucosamine sulfate group rat knee joints, ×200. (e) IHC quantitative analysis was shown as IOD (*n* = 3). ^*∗*^*p* < 0.05 compared with the blank control group, ^#^*p* < 0.05 compared with the Hulth model group. (a) Blank control group, (b) OA model group, (c) GBT recipe group, and (d) glucosamine sulfate group.

**Figure 4:** The localization of vimentin and DAPI was visualized under fluorescence microscopy after immunofluorescence staining. (a) Antivimentin antibody (green). (b) DAPI staining of nuclei (blue). (c) The merge of (a) and (b). Superficial markers of chondrocytes were detected using flow cytometry, with SW1353 cells as negative control. (d) 98% of chondrocytes show positive for type II collagen. (e) SW1353 cells show negative for type II collagen. (f) Type II collagen mRNA in chondrocytes and SW1353 cells was detected by qRT-PCR.

The article "Chondroprotective Effects of Gubitong Recipe via Inhibiting Excessive Mitophagy of Chondrocytes" was published in 2022. Journal: Evid Based Complement Alternat Med.

**Figure 5:** Effects of GBT recipe on chondrocytes viability. Chondrocytes were treated with different concentrations of GBT recipe (0, 50, 100, 150, 200, and 250 *μ*g/ml) for 12 h, and the viability of chondrocytes was assessed by the MTS assay; data are presented as mean ± standard deviation. (^*∗*^*p* < 0.05 compared with the blank control group).

**Figure 6:** Expression of MMP-13 in chondrocytes. Chondrocytes were pretreated with 50, 100, or 200 *μ*g/ml of GBT recipe for 1 hour and then stimulated with 100 ng/ml LPS for 12 h. (a) MMP-13 Western Blot band. (b) MMP-13 Western blot mean gray value. (c) MMP-13 mRNA expression. The data are derived from three independent experiments and expressed as the mean ± standard deviation. (^*∗*^*p* < 0.05 compared with the control group; ^#^*p* < 0.05 compared with the LPS-treated group).

**Figure 7:** Detection of mitophagy in chondrocytes using Mtphagy Dye (red). (a) Chondrocytes unstimulated control. (b) Chondrocytes stimulated with 100 ng/ml LPS for 12 h. (c) Chondrocytes pretreatment with 200 *μ*g/ml GBT recipe for 1 hour and then stimulated with 100 ng/ml LPS for 12 h. (d) Chondrocytes pretreatment with 100 nmol/ml DEX for 1 hour and then stimulated with 100 ng/ml LPS for 12 h.

**Figure 8:** Measurement of mitochondrial membrane potential (Δ*ψ*m) in chondrocytes using flow cytometric analysis after incubating with JC-1. P3 represents JC-1 red and P4 represents JC-1 green. (a) Chondrocyte unstimulated control. (b) 100 ng/ml LPS-stimulated chondrocyte for 12 h. (c) Chondrocyte pretreatment with 200 *μ*g/ml GBT recipe for 1 hour and then stimulated with 100 ng/ml LPS for 12 h. (d) Chondrocyte pretreatment with 100 nmol/ml DEX for 1 hour and then stimulated with 100 ng/ml LPS for 12 h. (e) The ratio of JC-1 green/red in each group; data are presented as mean ± standard deviation (^*∗*^*p* < 0.05 compared with the blank control group; ^#^*p* < 0.05 compared with the OA model group).

**Figure 9:** Expression of the ratio of LC3II and LC3I in mitochondria of chondrocytes, PINK1, and Parkin in chondrocytes. Chondrocytes were pretreated with 50, 100, or 200 *μ*g/ml of GBT recipe or 100 nmol/ml DEX for 1 hour and then stimulated with 100 ng/ml LPS for 12 h The data are derived from three independent experiments and expressed as the mean ± standard deviation (^*∗*^*p* < 0.05 compared with the control group; ^#^*p* < 0.05 compared with the LPS-treated group).

**Figure 10:** Expressions of PI3K, p-PI3K, AKT, and p-AKT in chondrocytes. Chondrocytes were pretreated with 50, 100, or 200 *μ*g/ml of GBT recipe or 100 nmol/ml DEX for 1 hour and then stimulated with 100 ng/ml LPS for 12 h. The data were derived from three independent experiments and expressed as mean ± standard deviation (^*∗*^*p* < 0.05 compared with the control group; ^#^*p* < 0.05 compared with the LPS-treated group).

The article "Chondroprotective Effects of Gubitong Recipe via Inhibiting Excessive Mitophagy of Chondrocytes" was published in 2022. Journal: Evid Based Complement Alternat Med.

**Table 1:** Information of primary antibodies.

Antibody	Manufacturer	Catalog no.	Molecular weights	Dilution	Electrophoretic gel concentration (%)
Anti-MMP-13	Abcam	ab39012	60 kD	WB 1 : 1000	10.0
Anti-AKT	Cell Signaling Technology	4691S	60 kD	WB 1 : 1000	10.0
Anti-phospho-AKT (Ser473)	Cell Signaling Technology	4060S	60 kD	WB 1 : 1000	10.0
Anti-Parkin	Santa Cruz	sc-32282	52 kD	WB 1 : 1000	10.0
Anti-PINK1	ABclonal	A11435	63 kD	WB 1 : 1000	10.0
Anti-LC3B	ABclonal	A19665	14 kD/16 kD	WB 1 : 1000	12.5
Anti-COX IV	ABclonal	A6564	17 kD	WB 1 : 1000	12.5
Anti-PI3K p85	ABclonal	A4992	85 kD	WB 1 : 1000	10.0
Anti-phospho-PI3K	Immunoway	YP0224	55 kD/85 kD	WB 1 : 1000	10.0
*β*-Actin	Zhongshan Jingqiao Biotechnology	TA-09	42 kD	WB 1 : 1000	10.0

**Table 2:** Chemical identification of GBT recipe.

No.	RT (min)	Name	Formula	Ion	Cal. m/z	Mea. m/z	Error (ppm)	MS/MS
1	2.39	Psoralen	C_11_H_6_O_3_	M−H	185.0244	185.0251	9.617	185.0251, 147.0325
2	5.52	Protocatechuic acid	C_7_H_6_O_4_	M − H	153.0193	153.0194	7.743	153.0194, 109.0296
3	6.09	Catechin	C_15_H_14_O_6_	M − H	289.0717	289.0717	3.582	289.0717
4	6.84	Pinoresinol diglucoside	C_32_H_42_O_16_	M + H	683.2545	683.2535	−3.167	519.1923, 357.2159
5	8.49	Sinomenine	C_19_H_23_NO_4_	M + H	330.1699	330.1709	2.772	330.1709
6	13.42	Epicatechin	C_22_H_18_O_10_	M − H	441.0827	441.0829	2.895	441.0829
7	15.77	Naringin	C_27_H_32_O_14_	M − H	579.1719	579.1722	2.328	579.1722, 271.0612, 151.0037
8	18.65	Tubeimoside I	C_63_H_98_O_29_	M + H	1319.627	1319.628	4.783	1319.628, 677.2439
9	19.19	Icariin	C_33_H_40_O_15_	M + H	677.2439	677.2439	3.822	677.2439, 369.1335, 313.0708

## Data Availability

The data supporting the findings of this study are available from the corresponding author upon request.
